The article "Evaluation Analysis of the Nephrotoxicity of Tripterygium wilfordii Preparations with CONSORT Harms Statement Based on Deep Learning" was retracted in 2023. Reasons: signs of a paper mill; suspected computer-generated content; unreliable results or conclusions; concerns about the data.

# Evaluation Analysis of the Nephrotoxicity of *Tripterygium wilfordii* Preparations with CONSORT Harms Statement Based on Deep Learning

**DOI:** 10.1155/2022/5054932

**Published:** 2022-04-07

**Authors:** Wuqiang Qi, Rui Chen, Minghui Chen, Meng Zhao, Mingzhao Wang

**Affiliations:** ^1^Pharmacy Department of Baojl, Hospital of Traditional Chinese Medicine, Baoji, Shaanxi 721001, China; ^2^Pharmacy Department of Hanzhong, People's Hospital, Hanzhong, Shaanxi 723000, China; ^3^Pharmacy Department of Xi'an, Central Hospital, Xi'an, Shaanxi 710003, China; ^4^Pharmacy Department of Affiliated Hospital of Shaanxi, University of Chinese Medicine, Xianyang, Shaanxi 712000, China

## Abstract

In this paper, the safety of *Tripterygium wilfordii* polyglycoside (TW) preparation was evaluated by combining literature research and evidence-based evaluation research, so as to provide evidence-based safety information of *Tripterygium wilfordii* polyglycoside preparation (nephroptosis) for government decision making and clinical application. In this paper, we propose a network structure inspired by the LSTM gate mechanism. All the research methods of the included references are evaluated by internationally recognized evaluation tools or standards. Prevalence was analyzed according to the type of intervention (e.g., time of administration) and route of administration. The results of this experiment provide methods and suggestions for the evaluation of traditional Chinese medicine nephroptosis in the future.

## 1. Introduction

Rehmannia glutinosa has the functions of promoting blood circulation and removing blood stasis, clearing heat and detoxification, eliminating swelling and knot, killing insects, and hemostasis and so on. Currently, there are a number of Chinese patent medicines containing Radix Rehmanniae ingredients approved for marketing by the State Food and Drug Administration (CFDA) [1]. These Radix Rehmanniae preparations are widely used as an immunosuppressant for the treatment. With its widespread use, its safety concerns have become increasingly prominent. Studies have shown that the most significant toxicity of tretinoin is reproductive toxicity and endocrine system and digestive system damage, in addition to nephroptosis, which is also a prominent toxic side effect of tretinoin. As early as the 1990s, there were case reports suggesting the nephroptosis of TW [2, 3]. In 2011, the UK Medicines Agency (MHRA) warned of the risk of serious side effects, including nephroptosis, and in April 2011, the CFDA warned of the toxic effects, and there were 839 cases of adverse reactions involving TW, of which renal insufficiency and renal failure were the more serious ones [4]. In contrast, a systematic evaluation/meta-analysis with secondary analysis of the available literature can provide an overall picture of the occurrence of adverse drug reactions.

The article "Evaluation Analysis of the Nephrotoxicity of Tripterygium wilfordii Preparations with CONSORT Harms Statement Based on Deep Learning" was retracted in 2023. Reasons: signs of a paper mill; suspected computer-generated content; unreliable results or conclusions; concerns about the data.

As early as the middle of the nineteenth century, scientists, having understood the internal structure of thujone, had decided to correlate the structure and properties of rhodopsin, hoping to predict the physicochemical properties of rhodopsin by the rules of the rhodopsin structure [5]. With the rapid development of theoretical and computational methods for regional descriptors, more and more statistical methods are being applied to the modelling process of compound property prediction [6–8]. The computational toxicology approach integrates the available data on the toxicity of thujone [9].

In terms of principle, toxicity prediction methods based on the structure of Rehmannia can be divided into three categories: read across [10], structural alerts (SAs) [11], and quantitative structure-toxicity relationships (QSTRs) [12]. The cross-referencing method is a method for predicting the endpoint information of a certain ragwort based on the known endpoint information of another ragwort with a similar structure. The theoretical basis of the method is constructed as follows: the physicochemical properties of a certain ragwort can be derived by analogy from a similarly structured ragwort. Also, this method saves unnecessary testing time by avoiding the need to test a large number of similar ragworts [13].

Since the 1970s, machine learning has evolved rapidly and researchers have explored different machine learning strategies and methods, expanding from single concept learning to multiple concept learning, focusing on combining multiple learning systems and applying them to various fields with great success. The most notable of these is the quantitative structure-activity relationship (QSAR) study [14]. The comprehensiveness and accuracy of data in data modelling are key to the success of the QSTR model. Ideally, toxicity data should be the result of the clinical performance of the drug, but this is a costly way to collect data and the amount of data is small. In vivo animal-based toxicity studies and in vitro cell and tissue-based toxicity studies can also provide more reliable toxicity data [15]. At present, some government and research institutions in the United States have joined forces to build a more authoritative database on the toxicity of TW, while countries and regions such as Europe and Japan have also established databases related to the safety of TW. In conclusion, the first step in establishing a QSTR model is to reasonably integrate and apply the existing toxicity data of TW, which requires researchers to reasonably integrate and summarize a large amount of data.

The article "Evaluation Analysis of the Nephrotoxicity of Tripterygium wilfordii Preparations with CONSORT Harms Statement Based on Deep Learning" was retracted in 2023. Reasons: signs of a paper mill; suspected computer-generated content; unreliable results or conclusions; concerns about the data.

The machine learning algorithm has certain advantages in dealing with problems such as large sample size and multi-dimension. Traditional machine learning algorithms include decision trees, random forests (RFs), support vector machines (SVMs), plain Bayesian, k-nearest neighbour methods, and so on [13].

## 2. Related Work

The kidneys, the main excretory organ of the chemistry, are particularly susceptible to the effects of drugs. Nephroptosis refers to drug-induced nephrotoxic reactions. Kleppe et al. [16] first reported two cases of acute renal failure after taking a Leigongteng tonic containing Guanmutong K. A Belgian study reported two cases of rapid progression of interstitial renal fibrosis to renal failure after taking a diet pill containing Fangqi and Houpu [17], and since then, the issue of Leigongteng nephroptosis has attracted widespread attention worldwide.

Our search revealed that the earliest reports of tretinoin nephroptosis from abroad appeared in the late 1980s, and the types of tretinoin and the types of nephroptosis reported varied. Gao et al. [18] reported a case of acute renal failure in a patient with back pain due to taking Radix Rehmanniae containing glycerolise acid. Wang et al. [19] reported a case of acute renal failure in a patient taking Radix Rehmanniae. Zhang et al. [20] reported 3 cases of interstitial renal damage caused by Angelica sinensis Siwei and Wuzhu Yusheng ginger decoction. Ioannidis [22] reported 1 case of acute renal failure due to the administration of 10 m1 of essential oil of Absinthium officials. Juszczak et al. [23] reported a case of rapid progression to end-stage renal failure after taking a formula containing aristocratic acid in Rehmannia. Moher et al. [23] reported a case of idiopathic acute interstitial renal fibrosis. The patient was treated with rehmannia tonic containing ginseng and Phellodendron. An animal study by Bwititi showed that cactus leaf extract caused an increase in urea nitrogen and creatinine concentrations and a decrease in serum Na + concentration.

In addition, the CFDA also reported the risk of nephroptosis of TW, including Shuanghuanglian injection and Qingkailing injection. The occurrence of adverse reactions to TW injection has a significant relationship with its unreasonable application, and the rational use of TW injection to reduce the occurrence of adverse reactions is still an important issue at this stage [24].

## 3. Construction of the Model

### 3.1. Modelling Data

According to the literature, the main factors affecting the efficiency of the model are the reliability of the original data, the data feature extraction method, modelling method, and the optimization strategy used [25]. In this study, our data were obtained from the most reliable Tox21 toxicity testing data available. All the structures in this dataset are given in SDF format, with the most basic and essential chemical information in the file. 6474 were inactive, and 1866 could not be determined to activate the ARE signalling pathway and were labelled as “active,” “inactive,” or “indeterminate,” respectively. To improve the accuracy of the model, we removed all the rhododendrons with the “uncertain” label. We downloaded 7668 species of ragweed from PubChem [7] based on the SIDs of all the ragweed species involved in the Tox21 challenge and processed them in the LigPrep module of the Schrodinger software [11], whose main procedures consisted mainly of converting the SDF files of small ragweed into 3D structures, hydrogenating each atom in the ragweed and removing ions and other mixed rhodopsin, and finally identifying and optimizing the conformation of small rhodopsin, for which we chose to delete those that had an irrational structure [2]. After these preprocessing procedures, 1136 active and 6299 inactive rhodopsin species remained. These regoliths were grouped into a training set, a test set, and an external validation set in a 4 : 1 : 1 ratio of the Kennard–Stone algorithm [3]. Notably, the grouping took into account both the similarity of the rigid structures and the self-organizing mapping (SOM) results.  Table 1 presents the grouping results for the datasets. The training set contains 4955 species of tripterygium, while the test set and external validation set both contain 1240 species of tripterygium.

The article "Evaluation Analysis of the Nephrotoxicity of Tripterygium wilfordii Preparations with CONSORT Harms Statement Based on Deep Learning" was retracted in 2023. Reasons: signs of a paper mill; suspected computer-generated content; unreliable results or conclusions; concerns about the data.

### 3.2. Calculation of the Lekomat Descriptor

In our approach, we use the DRAGON 7.0 [7] software to compute the descriptors. In fact, regolith descriptors play a very important role in model building, so we try to obtain as many regolith descriptors as possible. DRAGON 7.0 is a powerful descriptor calculation and analysis application that can calculate 5270 descriptors. Inevitably, given the structure of some of the smaller regoliths, there are some descriptors that cannot be calculated and the software sets them to default values. Considering the reliability of the data source, we removed all default values during the modelling process. That is, if there are default values in the data table, we remove the corresponding descriptors or small regoliths.

In addition, we calculated the fingerprint features (FPs) of the raffia. So-called FPs are a series of fixed-size Boolean vectors that encode the structural information of a regolith by decomposing its structure among all possible substructure patterns. With this method, the regolith is described as a series of binary strings based on its substructure. DRAGON 7.0 can compute two different types of fingerprints, namely, path fingerprints (PFPs) and extended connectivity fingerprints (ECFPs). We have chosen to compute ECFP features. For the SMARTS model, the corresponding position is set to “1” if a corresponding substructure exists in a given regolith. Otherwise, it is set to “0.” In this study, we used the DRAGON 7.0 software to obtain 1024 bit ECFPs for all small regoliths [5].

The article "Evaluation Analysis of the Nephrotoxicity of Tripterygium wilfordii Preparations with CONSORT Harms Statement Based on Deep Learning" was retracted in 2023. Reasons: signs of a paper mill; suspected computer-generated content; unreliable results or conclusions; concerns about the data.

Structural diversity of Ranunculus minor is essential for the construction of reliable global prediction models [6]. In this study, we performed a principal component analysis (PCA) for each of the two small rehmannia features [7]. This is shown in Figure 1. For the PCA results of the radio descriptors (Figure 1(a)), the toxic ratio (active) and non-toxic score (inactive) overlapped to a large extent. In contrast, for the PCA results of the fingerprint features (Figure 1(b)), both toxic ragwort and non-toxic ragwort were clustered in a smaller range and the dispersion of ragwort was small. In general, PCA scatter plots show whether or not [12] has a similar distribution of features in the feature space.

### 3.3. Highway Network

The depth of neural network models is currently deepening for applications in various fields. However, as the depth increases, deep neural networks are also exposed to the problem of gradient disappearance during training.

The inclusion of the highway network structure is very useful for training deep neural networks, and some studies have even been able to train neural networks with hundreds of layers without severe gradient disappearance [7].The highway network has shown powerful performance in a variety of applications, such as language modelling [4] and image classification [5]. Its structure is shown in Figure 2. The set input *x* is transformed through the network into an output. A normal neural network uses a nonlinear activation function to convert the input *x*. Here, the parameter bias is omitted from the equation for brevity of expression. Also, it not only is limited to representing the activation function but also can also be used to represent other operations of the neural network, such as convolutional and recurrent networks.

(1) $$\begin{array}{c} y=H\left(x,W_{H}\right). \end{array}$$

For the highway network neural network, two additional non-linear transformation layers are added, a transformation gate and a carry gate. In layman's terms, *T* represents the information obtained after the input information has been convolutional or recurrent, and *C* represents the part of the original input information *x* that is retained, of which T=sigmoid(*w*_*x*_+*b*). The first two parts represent the input into the gate unit, and the bottom part represents the input being copied directly into the final weighted summation operation [3].

(2) $$\begin{array}{c} y=H\left(x,W_{H}\right).T\left(x,W_{T}\right)+x.\text{C}\left(x,W_{c}\right). \end{array}$$

For ease of calculation, *C* = 1 − *T* is defined here.

(3) $$\begin{array}{c} y=H\left(x,W_{H}\right).T\left(x,W_{T}\right)+x.\left(1-T\left(x,W_{T}\right)\right). \end{array}$$

It is important to note that the dimensions of *x*, *y*, *H*, and *T* must be consistent. So, to ensure that the dimensions are consistent, either use subsampling or zero-padding strategies or use normal line layers to change the dimensionality to be consistent.

The article "Evaluation Analysis of the Nephrotoxicity of Tripterygium wilfordii Preparations with CONSORT Harms Statement Based on Deep Learning" was retracted in 2023. Reasons: signs of a paper mill; suspected computer-generated content; unreliable results or conclusions; concerns about the data.

## 4. Results and Discussion

### 4.1. Predictive Model Based on the Regulus Descriptor

In this study, we used DNN, HN, RNN, RF, and SVM algorithms to construct the ARE response prediction models based on the thunderclap descriptors. The statistical results of these models on the training set, test set, and validation set are shown in Table 2. In order to present the results of the models clearly, we have integrated and analyzed the result metrics for the training set, test set, and validation set, respectively, and presented them as radar plots. The height of all metrics will be represented by the size of the graphs in the radar plot. The area of the graph can also characterize the quality of the model. The larger the area of the graph constructed for each metric, the better the performance of the constructed model. The radar plot of the ARE toxicity prediction model based on the small thunderbolt descriptor feature is shown in Figure 3.

For the training set data, all models had high levels of SE, SP, MCC, F1-score, precision, and ACC. Notably, the SVM model showed a lower precision (0.596) and the DNN model exhibited a lower SE level (0.694). This could be attributed to the fact that there were fewer registers in the training set that could activate the ARE pathway. For both the test and validation sets, the indices of all models showed a similar trend, with all tending to predict thunderbolts as non-toxic thunderbolts. The main reason for this is the imbalance in the dataset, with fewer small regoliths able to activate the ARE pathway in both the test and validation sets. Of these models, the RNN model had the highest SE value, but the other metrics of the RNN model were not particularly impressive. Otherwise, the HN model had significantly higher SE values for all metrics than the other models, suggesting that the HN model has better predictive accuracy than the other models. In addition, ROC-AUC is critical to model performance, and all models are shown in Figure 4. Compared to the previous models, the DNN model we constructed based on the Raijin descriptor has higher ROC-AUC values and ACC values, indicating that our DNN model is more reliable.

The article "Evaluation Analysis of the Nephrotoxicity of Tripterygium wilfordii Preparations with CONSORT Harms Statement Based on Deep Learning" was retracted in 2023. Reasons: signs of a paper mill; suspected computer-generated content; unreliable results or conclusions; concerns about the data.

For the ROC-AUC metric, the DNN model outperformed the external validation set predictions for the ROC-AUC metric, while the HN exhibited a higher ACC (0.908) as well as a higher MCC (0.601) and F1-score (0.625) than the DNN. In the traditional machine learning method RF, SP (0.999) and precision (0.986) were relatively higher, and these metrics tended to classify the rhizomes as non-toxic rhizomes, possibly due to the unbalanced distribution of our dataset, but also reflecting the fact that the method may be relatively sensitive to the unbalanced distribution of positive and negative samples and prone to overfitting during modelling problems in the modelling process. In contrast, the RNN model exhibited a higher SE value (0.579) than the other models, suggesting that RNN may not be particularly sensitive to data imbalance problems, i.e., not prone to overfitting problems during the training process.

In this study, we used ROC-AUC as the main evaluation index and combined with other evaluation indexes for comprehensive evaluation. We found that the DNN had the best ROC-AUC results, and the other model metrics had better results. Therefore, the prediction performance of the DNN model based on the characteristics of the tripterygium descriptors was better than other models.

### 4.2. Fingerprint Characteristics of Tripterygium

In addition to the descriptors of ragwort, we also constructed toxicity prediction models for the ARE dataset based on ragwort fingerprint features.  Figure 5 illustrates the frequency of the 1024 typical fingerprint features in the dataset. The fingerprint features were used to construct six models including DNN, HN, RNN, CNN, RF, and SVM. The results are shown in Table 3, and the corresponding radar plots are shown in Figure 6.

For the training set, five of all six models performed very well, with only the RNN model showing relatively poor performance. The reason for the poor RNN results may be that the RNN excels at processing sequential information, whereas for the ARE response dataset, its sequential correlation for the thunderclap fingerprints may be less pronounced. In the test set results, SP, ACC, and precision values were relatively stable, while SE, F1-score, and MCC showed more variable results. The HN model showed the highest SE value (0.611), while SVM showed the lowest SE value (0.289). For the external validation set, the SE value of HN (0.626) performed better than the other models, indicating that the HN model has better predictive power.

The article "Evaluation Analysis of the Nephrotoxicity of Tripterygium wilfordii Preparations with CONSORT Harms Statement Based on Deep Learning" was retracted in 2023. Reasons: signs of a paper mill; suspected computer-generated content; unreliable results or conclusions; concerns about the data.

The ROC-AUC curves of the modelling results based on the tripterygium fingerprint features are shown in Figure 7, with all six models showing better ROC curves and higher ROC-AUC. Models based on [12] fingerprint features have better results compared to the models based on [12] descriptors. It is worth noting that the RF model based on the tripterygium fingerprint features has the highest ROC-AUC (0.924), even better than the corresponding DNN model (0.917). However, the ROC-AUC result for RF was not significantly superior to 0.007, so we integrated the other model result metrics and found that the DNN model had an overall higher and more stable result metric, suggesting better performance of the DNN model.

As the results from the external validation set show, deep learning has better generalization capabilities. By comparing the results based on different results of different modelling approaches based on different tripterygium features, we found that the validity of the model based on tripterygium fingerprint features far exceeded that of the model based on tripterygium descriptors. It was clear that the fingerprint features of tripterygium showed better modelling performance than tripterygium descriptors in ARE toxicity prediction. Therefore, the fingerprint features of Ranunculus minor may be a guide for subsequent studies.

Compared to traditional machine learning methods, deep learning has better learning capabilities and deep learning algorithms can extract high-level features of the data. For the descriptor-based models, DNN showed the highest ROC_AUC and ACC, while HN showed the best SE results. The results of modelling based on the fingerprint features of thunderbird show that the DNN model still performs well, while the HN shows higher SE than the other models. In addition, we can use the RNN and CNN algorithms, which have not been previously attempted for thunderbird modelling, to build reliable predictive models for thunderbird performance. Furthermore, CNN and RNN can extract higher dimensional and deeper serial relationship features for future data analysis.

## 5. Conclusions

*Rehmannia glutinosa* has the effects of promoting blood circulation and removing blood stasis, clearing heat and detoxification, eliminating swelling and knot, killing insects and hemostasis. However, the effective analysis of its yellow component is the pain point of Chinese patent medicine research. Inspired by the gating mechanism of LSTM, this paper proposes a network structure. Through this structure, the internationally recognized evaluation tools or standards evaluate the methodological quality contained in the study and analyze the intervention type, administration route, administration time, and study type of drugs. Compared with other models, our method has the highest SE value.

The article "Evaluation Analysis of the Nephrotoxicity of Tripterygium wilfordii Preparations with CONSORT Harms Statement Based on Deep Learning" was retracted in 2023. Reasons: signs of a paper mill; suspected computer-generated content; unreliable results or conclusions; concerns about the data.

## Figures and Tables

**Figure 1:** Plot of PCA of the tripterygium features.

**Figure 2:** Internal diagram of the highway network model.

**Figure 3:** Radar plot of the classification model constructed based on the Raijin descriptor features.

**Figure 4:** ROC diagram of the model based on the Raijin descriptor features (test set on the left and the external validation set on the right).

**Figure 5:** Frequencies corresponding to the fingerprint features.

**Figure 6:** Radar plots of modelling results based on the fingerprint features of the thunderbolt.

**Figure 7:** ROC plots of the model based on the fingerprint features of tripterygium.

**Table 1:** Statistics for the ARE dataset.

Group	Training set	Test set	External validation set
Activation	756	190	190
Inactivation	4199	1050	1050

**Table 2:** Results of modelling based on the characteristics of the rayado descriptors.

Methods	RF			SVM			DNN			HN			RNN		
Group	Tr	Tst	Val	Tr	Tst	Val	Tr	Tst	Val	Tr	Tst	Val	Tr	Tst	Val

F1	0.96	0.56	0.55	0.74	0.46	0.51	0.79	0.55	0.49	0.95	0.66	0.62	0.92	0.60	0.54

**Table 3:** Modelling results based on the fingerprint characteristics of the Leihmannia.

Methods	RF			SVM			DNN			HN			RNN		
Group	Tr	Tst	Val	Tr	Tst	Val	Tr	Tst	Val	Tr	Tst	Val	Tr	Tst	Val

F1	0.97	0.62	0.61	0.97	0.43	0.46	0.97	0.70	0.70	0.97	0.68	0.70	0.89	0.66	0.60

## Data Availability

The data used to support the findings of this study cannot be shared due to trade confidentiality.
